# Prognostic Diagnosis for Breast Cancer Patients Using Probabilistic Bayesian Classification

This article has been retracted.

**DOI:** 10.1155/2022/1859222

**Published:** 2022-07-25

**Authors:** N. Junath, Alok Bharadwaj, Sachin Tyagi, Kalpana Sengar, Mohammad Najmus Saquib Hasan, M. Jayasudha

**Affiliations:** ^1^The University of Technology and Applied Science Ibri Sultanate of Oman, Oman; ^2^Department of Biotechnology, GLA University, Mathura, India; ^3^Bharat Institute of Technology, School of Pharmacy Meerut, India; ^4^Biosense Lifecare Research and Development Laboratory, Kalphelix Biotechnologies, Kanpur 208011, India; ^5^Wollega University, Nek'emtē, Ethiopia; ^6^School of Computer Science and Engineering, Vellore Institute of Technology, Chennai, India

## Abstract

The diagnosis and treatment of patients in the healthcare industry are greatly aided by data analytics. Massive amounts of data should be handled using machine learning approaches to provide tools for prediction and categorization to support practitioner decision-making. Based on the kind of tumor, disorders like breast cancer can be categorized. The difficulties associated with evaluating vast amounts of data should be overcome by discovering an efficient method for categorization. Based on the Bayesian method, we analyzed the influence of clinic pathological indicators on the prognosis and survival rate of breast cancer patients and compared the local resection value directly using the lymph node ratio (LNR) and the overall value using the LNR differences in effect between estimates. Logistic regression was used to estimate the overall LNR of patients. After that, a probabilistic Bayesian classifier-based dynamic regression model for prognosis analysis is built to capture the dynamic effect of multiple clinic pathological markers on patient prognosis. The dynamic regression model employing the total estimated value of LNR had the best fitting impact on the data, according to the simulation findings. In comparison to other models, this model has the greatest overall survival forecast accuracy. These prognostic techniques shed light on the nodal survival and status particular to the patient. Additionally, the framework is flexible and may be used with various cancer types and datasets.

## 1. Introduction

Breast cancer is the one of most common malignant tumors in women in my nation and the sixth-largest cause of cancer-related mortality [1]. Breast cancer incidence and death among Chinese women have been rising fast in recent years, with certain places seeing considerable and rapid increases [2, 3]. To minimize patient mortality, researchers must study and select more effective treatment plans, or design specific treatment plans for patients, both of which rely on accurate prognostic analysis and patient survival prediction.

Based on one or more predictor variables, the logistic method is used to predict the class (or category) of persons (x). It is used to simulate a binary result, or a variable with only two potential values, such as 0 or 1, yes or no, or sick or not. The main goal of using logistic regression analysis is to make sure that it is the best analytical form that can assign data to groups when the dependent variable in various scientific domains has two or more levels and the control variables are both discontinuous and continuous. Whereas by microscopic inspection of suspicious tissue that has been removed via biopsy or surgical resection, the histological type is identified. If the tissue under examination exhibits a different histological type than what is typically seen there, it may indicate that the cancer is spreading there from a primary location. Medical students benefit much from studying histology in a variety of ways. It aids students in comprehending how tissues and cells are arranged in a typical organ system. Additionally, it links the development of different tissues to each function, which links structure to function.

In the study of the prognostic factors of cancer, the researchers found that there are many factors affecting the prognostic level of patients, and they can be roughly divided into the following three categories: First, the demographic and genetic characteristics of patients, such as the incidence of patients' age and whether they carry breast cancer susceptibility genes; second, disease characteristics, such as tumor location, size, and histological grade; third, treatment options, such as chemotherapy and immunotherapy [4]. At present, a large number of statistical methods have been analyzed and studied on the above factors, to quantify the influence of these factors on the prognosis of patients [5, 6]. The Bayesian method gives no instructions on how to choose a precedent. The selection of a previous can be done in any method. The ability to convert irrational prior beliefs into mathematically specified prior is necessary for Bayesian findings. Without exercising caution, you might produce false findings. It may result in posterior distributions with strong previous impact. Practically speaking, it could occasionally be challenging to persuade subject-matter experts who disagree with the accuracy of the selected prior. It frequently has a significant computational cost, particularly in models with several parameter choices. In addition, if a different random seed is used, simulations provide somewhat different results. It should be noted that minor deviations in simulation results do not refute the initial assertion that Bayesian judgments are precise. Given the log-likelihood and the priors, the posterior distributions of a parameter are accurate; however, simulation-based estimations of the posterior numbers might vary depending on the random number employed in the methods.

The first step in the prognostic analysis is to determine which factors have the most significant effect. Among the various factors listed above, some factors are highly correlated or even redundant and cannot provide more information. Since the follow-up investigation of the patient's prognosis requires a lot of time and economic cost, the first step in establishing a survival prediction model is to select significant prediction features to make the prediction model as concise as possible, that is, under the premise of obtaining almost the same amount of information, select the model with the least amount of features. At present, the commonly used feature selection methods include forward feature selection, reverse feature selection, or the use regression model for univariate analysis to select features with greater influence weights. In this paper, after referring to a large number of literature and comparing the advantages and disadvantages of various feature selection methods [7, 8], the commonly used reverse feature selection method is selected, and the most significant factors are selected for prognostic analysis, of which LNR is one of the most significant disease-characterizing factors. Recent research suggests that LNR, as opposed to the number of positive nodes alone, is better good at predicting overall survival and relapse survival rate. It is regarded as a significant prognostic factor in the gastrointestinal system, breast, bladder, and pancreatic cancers. LNR has been found to have a stronger predictive value than the lymph node phase. Due to its simplicity and repeatability, LNR can be used in the follow-up of many cancers. There has not been established a unified and widely accepted appropriate cut-point for LNR despite numerous studies on epithelial malignancies. Divergences may be caused by variations in sample sizes, inclusion requirements, disease kinds, assessment criteria, and statistical techniques.

LNR is one of the most important variables in cancer prognosis analysis, especially for recurrence risk. This trait improves cancer prognosis and survival rate. Author [9] discovered that the metastatic lymph node ratio predicts survival in cervical squamous cell carcinoma patients. The author used LNR and other parameters to use the standard Bayesian model to predict pancreatic cancer patient's survival rate and survival rate [4]. The author analyzed 2591 Sun Yat-sen University Cancer Center medical data from 1998 to 2007 using a standard regression model and found that breast cancer patients with lower LNR levels were more likely to have breast cancer. LNR predicts overall, disease-free, and metastasis-free survival [10].

LNR utilizes the number of positive lymph nodes on a slide divided by the total number seen. The test's LNR result may differ greatly from the patient's real LNR. Total lymph nodes in the test sample are simply a local observation. This causes a substantial difference between the experimental LNR and the patient's real LNR. More lymph nodes identified during slice identification means a more accurate LNR value. The LNR test result obtained from total identified lymph nodes and positive lymph nodes is an approximation of the patient's genuine LNR [4]. In this work, extra pathological characteristics were incorporated to enhance LNR estimation accuracy, and the LNR value was calculated using the logistic regression technique to provide a closer assessment of the patient's total LNR. In this paper's simulation, the overall LNR estimate based on logistic regression and the LNR local cutoff value were compared on prognostic analysis.

As mentioned previously, the overall estimates of LNR based on logistic regression models are important clinical features for prognostic analysis. At present, the classical regression model is widely used in prognostic analysis to predict the survival rate of patients. This model was proposed by a British statistician in 1972 [11], and its basic idea is to express the survival rate of patients as a risk function, that is, the probability of death of an individual in a certain unit of time during the survival process. The regression model is a semiparametric survival analysis model [12].

Compared with the parametric model [13], its conditions are more relaxed, and the survival data does not need to meet a certain distribution in advance. Compared with the parametric model, its test efficiency is relatively higher, and the survival function and the benchmark risk function can be obtained at the same time when the survival distribution and benchmark risk function of the data are unknown. It is these advantages that make the classic regression model popular and widely used in the decades after it was proposed. However, in a classic regression model, the covariate coefficients are always constant and cannot reflect the dynamic effects of predictors on survival over time [14]. By combining the prior knowledge of each parameter and the observation data, the posterior distribution of the parameters was inferred and continuously updated, to better capture the prediction variables in different time intervals' effect on survival.

Figure 1 shows this study's flowchart. First, SEER samples were selected (The Surveillance, Epidemiology, and End Results). 20-80-year-old women with breast cancer and at least one lymph node diagnosed between 2010 and 2012. Due to differences in overall survival rates across breast cancer subtypes [15], this investigation included only “Her2-/HR+” patients. 4,402 samples were obtained after screening.  Table 1 lists the samples. The leftover features are utilized for survival analysis after LNR features are chosen via reverse feature selection. Total lymph nodes, number of positive lymph nodes, M stage, and N stage have the greatest relationship with LNR, according to the Akaike Information Criterion (AIC) index. These are utilized to train a logistic regression model and estimate the LNR value. In the prognostic study, a dynamic Bayesian regression model was created to predict patient survival using overall LNR estimates as well as patient age, tumor size, and T stage.

### 1.1. Implications of Machine Learning in Breast Cancer Detection

Cancer has been described as a diverse illness with a wide range of subgroups. Early cancer diagnosis and prognosis are essential for clinical patient treatment, which has become a requirement in cancer research. Numerous research teams from the biomedical and bioinformatics fields have studied the use of machine learning (ML) techniques due to the significance of classifying cancer sufferers into high- or low-risk categories. These methods have been applied to stimulate the development and management of malignant diseases.

Furthermore, their significance is demonstrated by the fact that ML algorithms can recognize important characteristics in complicated datasets. Artificial Neural Networks (ANNs), Bayesian Networks (BNs), Support Vector Machines (SVMs), and Decision Trees (DTs) are a few of the methods that have been widely used in cancer research to construct prediction models that enable precise and effective decision-making. Although using ML techniques can enhance our comprehension of how cancer progresses, further validation is required before these techniques can be used in routine clinical practice. The author et al. did a comparative analysis of breast cancer detection using machine learning and biosensors. They found that automation is required since ML and biosensors are required to detect tumors from microscopic pictures. The goal of ML is to help computers learn for themselves. It is built on pattern recognition in observed data and creating models to anticipate outcomes rather than depending on specific pre-programmed rules and models [16]. The author et al. concluded that the most effective algorithm for detecting breast cancer is XGboost, which has a 98.24 percent effectiveness rate. The dataset must first be processed, though, before the method can be executed [17].

## 2. Data and Methods

### 2.1. LNR Estimation Based on Logistic Regression Model

LNR is computed by dividing the number of positive lymph nodes on a slice by the total number of lymph nodes. In reality, it is difficult to adequately depict the patient's total LNR by the LNR local resection value. This research evaluated additional relevant pathological information of LNR patients and used a logistic regression model to predict total LNR values. First, the LNR local cut value is used as the response feature, and the relevant pathological features are selected as input features through reverse feature selection. Then, the covariate coefficient is calculated by fitting the logistic regression model, and the patient's overall LNR is estimated using the covariate coefficient value.

The logistic regression model is a commonly used machine learning model, its form is relatively simple and intuitive, and it has good interpretability. In this paper, the regression analysis is performed using the range of the logistic regression model in the range of [0,1] to estimate the overall value of LNR within the same range. In this study, the basic form of the logistic regression model is as follows: for sample I, its response value, that is, the LNR value is Yi; 4 pathological features related to LNR are screened out through reverse feature selection as input features, which are positive lymph nodes, respectively. The number *X*_1_ is the total number of lymph nodes *X*_2_, the M stage *X*_3__,_ and the N stage *X*_4_. According to the logistic regression model, the relationship between the LNR value *Y*_*i*_ of sample I and its corresponding predicted feature *X*_*i*_ is:

(1) $$\begin{array}{c} y_{i}=\frac{1}{1+\exp\left[-\left(\beta_{0}+\beta_{1}X_{i,1}+∙∙∙∙∙∙∙+\beta_{1}X_{i,4}\right)\right]}=\frac{1}{1+\exp\left(-\beta^{T}X_{i}\right)}. \end{array}$$

Among them, *β*_0_ is a constant term, *β*_1_, *β*_2_, *β*_3_, and *β*_4_ are the covariate coefficients corresponding to each prediction feature, and *β* is a vector composed of the above covariate coefficients. *X*_*i*,1_, *X*_*i*,2_, *X*_*i*,3_, and *X*_*i*,4_ are the four predic eigenvalues sample m IIe I, and *X*_*i*_ is a vector composed of the above pride eigenvalues. After fitting the logistic regression model with the training set data, the covariate coefficients *β* corresponding to all the predicted features are obtained. After that, according to the coefficient *β* and the prediction feature *X*_*i*_, substituting Equation (1) can get the overall estimated value of LNR.

### 2.2. Probabilistic Bayesian-Based Dynamic Regression Model

The basic form of the classic regression model is:

(2) $$\begin{array}{c} \lambda \left(t\;|\;Z\right)=\lambda_{0}\left(t\right)\exp\left\{Z^{T}\beta_{s}\right\}. \end{array}$$

The covariate coefficients in a standard regression model stay constant across time points. In practice, however, the effect of each predictor on patient survival is frequently time-varying. To this aim, the Bayesian dynamic regression model encodes the covariate coefficients at different time points as *s*(*t*), and the posterior distribution is calculated using the Bayesian approach and the survival data. Wang et al. devised this approach, which is only briefly described in this work.

The dynamic regression model based on the Bayesian technique takes the following basic form:

(3) $$\begin{array}{c} \lambda \left(t\;|\;Z\right)=\lambda_{0}\left(t\right)\exp\left\{Z^{T}\beta_{s}\left(t\right)\right\}, \end{array}$$

where *Z* is the matrix of predictors for all samples, *λ*_0_(*t*) is the baseline risk at time *t*, and *β*_s_(*t*) is the vector of covariate coefficients at time *t*. In this dynamic model, both *λ*_0_(*t*) and *β*_*s*_(*t*) are assumed to be left-continuous step functions. The reference risk function must be estimated in the model *λ*_0_(*t*) and the covariate coefficient vector *β*_*s*_(*t*) specific step times and corresponding step values and step time points to accomplish the goal of dynamic parameter estimation Let: Θ = {ln*λ*_0_(*t*), *β*_*s*_(*t*); *t* > 0}, All unknown parameters are included in the set., use *θ*(*t*) to refer to ln *λ*_0_(*t*) or *β*_*s*_(*t*) in an amount.

All unknown parameters are estimated from data samples. For sample *i*(*i* = 1, 2, ⋯, *n*), let *T*_*i*_ denote the time at which the event “patient death” occurred. If *T*_*i*_ is known, the sample data is complete survival data. If only *T*_*i*_ ∈ [*L*_*i*_, *R*_*i*_) can be determined and *R*_*i*_ is a finite value, the sample data is interval-censored; if *R*_*i*_ = ∞, the sample data is right-censored. Let Δ*k* = *SK* − *SK*_−1_ represent the width of the *k*^th^ grid interval, and count *λ*_*k*_ = *λ*_0_(*SK*), *β*_*k*_ = *β*(*SK*). Finally, let *Dobs* = {*Ti* ∈ [*Li*, *Ri*), *Zi*; *i* = 1, 2, ⋯, *n*}; this set represents the survival information of all samples and the information of the predictor variables related to the survival analysis.

In dynamic models, a Bayesian approach as:

(4) $$\begin{array}{c} \left(\text{o}\;|\;x\right)=p\left(\text{o}\right)\frac{p\left(x\;|\;\text{o}\right)}{p\left(x\right)}\propto p\left(\text{o}\right)L\left(x\;|\;\text{o}\right). \end{array}$$

This formula says that the posterior distribution of the parameters is proportional to the product of the joint prior distribution *p*(*o*) of the parameters and the sample likelihood *L*(*x* | *o*). Among them, the sample likelihood *L*(*x* | *o*) can be expressed as

(5) $$\begin{array}{c} \left(x\;|\;o\right)=\overset{N}{\underset{i=1}{\prod }}\mathrm{Pr}\left(T_{i}\in \left[L_{i},R_{i}\right)\;|\;\text{o},{xZ}_{i}\right), \end{array}$$

where *n* is the total number of samples. The likelihood contribution of any one of the samples *i* is:

(6) $$\begin{array}{c} \mathrm{Pr}\left(T_{i}\in \left[L_{i},R_{i}\right)\;|\;o,x_{i}\right)=\mathrm{Pr}\left(T_{i}>L_{i}\;|\;o,x_{i}\right)-\mathrm{Pr}\left(T_{i}>R_{i}\;|\;o,x_{i}\right). \end{array}$$

In

(7) $$\begin{array}{c} P\text{r}\left(T_{i}>t\;|\;o,x_{i}\right)=\exp\left\{-\overset{K}{\underset{k=1}{\sum }}I\left(s_{k}<t\right)\Delta_{k}\lambda_{k}\exp\left(x_{i}^{T}B_{k}\right.\right\}, \end{array}$$

*I*(•) is the indicator function in the preceding formula; if • is true, *I*(•) = 1, else *I*(•) = 0.

(8) $$\begin{array}{c} \left\{\begin{array}{c} \begin{array}{c} \theta \left(\tau_{1}\right)\;|\;\omega \sim N\left(0,c\omega \right)\\ \theta \left(\tau_{j}\;|\;\theta \left(\tau_{j-1}\right),\omega \sim N\left(\theta \left(\tau_{j-1}\right),\omega \right.\right),j=2,3,\cdots ,J\\ \omega \sim \text{Inverse Gamma}\left(\alpha ,n\right) \end{array} \end{array}\right.. \end{array}$$

The prior distribution hypothesis for that parameter at the preceding time interval is connected to the prior distribution hypothesis for the covariate coefficients for each period. The link between the previous distribution assumptions for the parameters is shown in Figure 2. The circular box's parameters are predetermined constants, and the box's parameters only know which distribution they follow; therefore, the particular value must be approximated.

The joint prior distribution of*θ*(*t*) and*ω*, *π*(*θ*(*t*), *ω*)is proportional to the following formula, according to the dynamic prior connection of the Bayesian framework and parameters given earlier: The joint prior distribution of*θ*(*t*) and*ω*, *π*(*θ*(*t*), *ω*)is proportional to the following formula: dynamic prior connection of the Bayesian framework and parameters indicated earlier.

(9) $$\begin{array}{c} \text{alaomegala}\frac{\eta^{\alpha }}{\Gamma \left(\alpha \right)}\omega^{-\alpha -1}\exp\left(-\frac{\eta }{\omega }\right)\omega^{-j/2}\;\exp\left\{-\frac{\theta {\tau_{1}}^{2}}{2c\omega }\right\}\underset{j>2}{\prod }\exp\left\{-\frac{{\left[\theta \left(\tau_{j}\right)-\theta \left(\tau_{j-1}\right)\right]}^{2}}{2\omega }\right\}. \end{array}$$

(*η*^*α*^/Γ(*α*))*ω*^−*α*−1^exp(−*η*/*ω*) is the probability density function of *ω*, where the remainder is the product of the probability density functions of *θ*(*τ*1), *θ*(*τ*2), ⋯, *θ*(*τJ*). For each *θ*(*t*), there is its corresponding *ω*. The joint probability density of Θ and *ω* can be obtained by multiplying *p* + 1 by Equation (9). Equations (5), (8), and (9) may be used to compute the posterior component of all parameters (9). The posterior distribution, however, cannot be determined directly owing to the complicated shape of the joint probability density Θ and *ω*. The posterior distribution is calculated using Gibbs Sampling for this purpose.

## 3. Simulation Results

For data processing and analysis, R Studio 1.0.143 was utilized, and the R language version used was 3.4.4, with 4402 samples screened in SEER. These samples are randomly separated into training and test sets throughout the simulation. The test set has 1402 samples, whereas the training set contains 3000 samples.

### 3.1. LNR Estimation

The number of positive lymph nodes, the total number of lymph nodes, the M stage, and the N stage were all utilized to determine the LNR value after reverse feature selection. The logistic regression model obtained the lowest AIC value in 1968 when these four characteristics were used. A low AIC score means the model can fit the data well with fewer parameters.  Table 2 shows the covariate coefficients of certain predicted characteristics after logistic regression model training. The standard deviation of the two characteristics of a total number of lymph nodes and several positive lymph nodes is the lowest in the table, suggesting that these two characteristics have the strongest link with LNR.

To judge whether there is an overfitting problem, the MSE of the training set and the test set data after fitting the logistic probability regression model are calculated, respectively. After calculation, the MSE value of the training set data after fitting the model is 0.019, and the MSE value of the test set data is 0.021. The two are on the same order of magnitude and the gap is small. According to this judgment, the logistic probability regression model after training has no overfitting phenomenon. In the subsequent calculation process, it is feasible to use the LNR value estimated by this model.  Figure 3 shows the predicted training and test set standard deviation coefficients.

### 3.2. Subsistence Analysis

To test the predictive effect of the overall estimate of LNR on patient survival, two datasets were used in this study in the survival analysis section. Both contain patient survival information, T and N stage information, age at diagnosis, and tumor size; the only difference is that dataset 1 uses LNR local resection values and dataset 2 uses LNR overall estimates. Furthermore, so that the dynamic regression model based on the Bayesian method can better reflect the influence of predictors on the survival rate of patients at different time stages, this paper uses the classical regression model and the dynamic regression model, respectively. Therefore, different datasets were paired with different survival analysis models, resulting in a total of 4 model models to compare the difference in results between them. The main features of the four models are shown in Table 3. All models were set to 500 Gibbs samples.

In this paper, the Log Pseudo Marginal Likelihood (LPML) is used as the evaluation index of the survival analysis model. For the model, the larger the value of this indicator is, the more the sample supports the model. The LPML values of the four models are -719.45, -705.81, -703.11, and -694.43. As shown in Table 3, the LPML value of Model_2 is larger than that of Model_1. Likewise, the LPML value of Model_4 is greater than the LPML value of Model_3. Based on this numerical comparison, it can be seen that using the LNR overall estimate has a relatively good model fit. Also, the LPML values of Model_3 and Model_4 are higher than those of Model_1 and Model_2. This result shows that the dynamic regression model based on the Bayesian method can better fit the survival data than the classical regression model.

To judge the effect of the model more intuitively, the overall survival rate-time curves obtained by analyzing the training set and test set data of the four models were drawn. In comparison, the overall survival rate-time curve of patients was drawn using the Kaplan-Meier method (hereinafter referred to as the KM method). It is closer to the KM curve, indicating that the prediction effect of the model is relatively better. Shown in Figure 4 are the survival-time curves for the training and test set data predicted by the four models. As can be seen from the figure, Model_1 and Model_2 using the classical regression model perform worse than Model_3 and Model_4 using the dynamic model on both the training set and the test set. The overall survival-time curve predicted by the dynamic model is closer to reality. In addition, the curves obtained by Model_3 and Model_4 on the training set and test set are relatively close, but it can still be seen that the Model_4 curve has a relatively good prediction effect, and Model_4 has a lower LPML value. This suggests that the survival-time characteristic curve can be more accurately predicted using the overall estimate of LNR.

## 4. Conclusion

This paper points out two important problems in breast cancer prognosis analysis and proposes corresponding solutions: one is that the LNR value obtained by the experimental detection is greatly affected by the observation error, which has deviations in the subsequent survival analysis process; regression models were unable to capture the dynamic effects of cancer-related factors on patient survival across time intervals. For the first question, this study first used logistic regression to estimate the LNR population value and then used the LNR population estimate value with other predictor variable information and survival data to fit a Bayesian method-based dynamic regression model. Compared with the use of LNR local cutoff values, the use of estimated values reduces the effect of the smaller total number of lymph node tests on the LNR value, as well as the effect of individual differences between patients on the LNR value. For the second problem, using the dynamic regression model based on the Bayesian method can better capture the impact of different time stages and predict the impact of characteristics on the survival rate of patients; The Bayesian method of the empirical distribution predicts the parameters more accurate.

The data set used in this article is part of the data of female breast cancer patients in SEER, and the algorithm is implemented using R language. To verify the performance of the method described in the paper, LPML values are used as a measure of model performance. Simulation results show that the model using the LNR estimate and the Bayesian-based dynamic regression method has the highest LPML value, indicating that the data best supports the model. In addition, to verify the prediction effect of the model, the survival rate-time curve of the test set data was calculated using the KM method and used as a benchmark, which was compared with that predicted by the logistic regression model to estimate LNR and the dynamic survival analysis model based on the Bayesian method. Survival-time curves were compared. The results show that the two curves have many overlaps, and the trends are consistent. In future research, we can continue to explore the predictive effect of LNR on the survival rate of cancer patients, and try to use other machine learning methods, such as decision trees and random forests, to estimate the LNR value. The predictive value of the lymph node ratio (LNR), which is measured as the percentage of positive nodes tested, has attracted attention more lately. However, there are not enough statistical techniques to model LNR and its impact on cancer survival together. T and M stages as well as histologic grade were significantly predictive of LNR status. Age, gender, marital status, grade, histology, T and M stages, tumor size, and radiation treatment were all significant predictors of survival. An extremely significant, nonlinear influence of LNR on survival was discovered. Furthermore, the survival model's prediction ability outperformed that of studies using predictors with more customized and uniform patient populations. The understanding and management of illness rely heavily on prognostic models. These prognostic techniques shed light on the nodal survival and status particular to the patient. Additionally, the framework is flexible and may be used with various cancer types and datasets.

The probabilistic technique has the benefit of allowing current models to be expanded with previous information. This may be done at both the structural and parameter levels. This will have an effect on the variables that appear in the Markov blanket, resulting in an attribute selection approach based on data and previous biological knowledge, with automated tweaking of the data-prior knowledge balance. Furthermore, because Bayesian networks are not tailored for classification and instead provide a more generic framework by modeling a multidimensional probability distribution; the claimed performance may be improved by employing more traditional classifiers. We are now researching the usage of Bayesian networks as feature selectors, accompanied by Least Squares Support Vector Machines for classification.

## Figures and Tables

**Figure 1:** Overall flowchart.

**Figure 2:** Prerelationship between parameters.

**Figure 3:** Predicted training and test set standard deviation coefficients.

**Figure 4:** Predicted training and test set survival-time curves.

**Table 1:** Dataset sample characteristics.

Feature name	Value	Number of samples (percentage)	Mean
Track time	0~59	4405 (100)	37.89
State	Die	160 (3.8)	
	Survive	4250 (95.69)	
Total number of lymph nodes	1~84	4405 (100)	12.68
Number of positive lymph nodes	1~82	4405 (100)	4.71
Age at diagnosis	20~80	4405 (100)	57.12
	[20,30)	48 (1.3)	
	[30,40)	334 (8.6)	
	[40,50)	951 (26.34)	
	[50,60)	1064 (28.26)	
	[60,70)	975 (25.18)	
	[70,80]	520 (13.25)	
T stage	T0	78 (1.9)	
	T1	1028 (32.8)	
	T2	1766 (40.4)	
	T3	600 (13.8)	
	T4	235 (5.6)	
	TX adjusted	58 (1.4)	
	Others	240 (5.5)	
M stage	M0	4112 (94.12)	
	M1	240 (5.6)	
	M2	53 (1.4)	
N stage	N1	2870 (65.4)	
	N2	889 (20.11)	
	N3	588 (13.6)	
	NX adjusted	58 (1.2)	

**Table 2:** Coefficients of some predictors.

Predictor variable	Estimated value	Standard deviation
Intercept	0.227	0.084
Total number of lymph nodes	-0.183	0.015
Number of positive lymph nodes	0.367	0.029
M1	0.589	0.248
MX	-0.148	1.245
N2	0.505	0.141
N3	0.531	0.248
NX adjusted	0.298	0.173

**Table 3:** Model features.

Name	LNR data	Survival analysis model	LPML
Model_1	Local cut value	Standard model	-719.45
Model_2	Overall estimate	Standard model	-705.81
Model_3	Local cut value	Dynamic model	-703.11
Model_4	Overall estimate	Dynamic model	-694.43

## Data Availability

The data shall be made available on request.
